# Thermally-stable single-atom catalysts and beyond: A perspective

**DOI:** 10.3389/fchem.2022.959525

**Published:** 2022-07-14

**Authors:** Sixu Liu, Jiwei Li, Haifeng Xiong

**Affiliations:** ^1^ State Key Laboratory of Physical Chemistry of Solid Surfaces, College of Chemistry and Chemical Engineering, Xiamen University, Xiamen, China; ^2^ Innovation Laboratory for Sciences and Technologies of Energy Materials of Fujian Province (IKKEM), Xiamen, China

**Keywords:** single-atom catalysts, thermally stable, atom trapping, metal-support interaction, vapor-phase self-assembly

## Abstract

Single-atom catalysis is a research Frontier and has attracted extensive interests in catalysis. Significant progresses have been carried out in the synthesis and characterization of metal single-atom catalysts (SACs). However, the stability and catalytic reactivity of metal SAC at elevated temperatures are not well documented because single atoms sinter at elevated temperatures. Therefore, the development of stable and reactive SAC at high temperatures remains a formidable challenge. In this perspective, we summarize recent efforts on the preparation of the thermally-stable SACs synthesized at elevated temperature *via* the reverse-Ostwald ripening mechanism, including the approaches of atom trapping and vapor-phase self-assembly. The reducibility of lattice oxygen, the loading upper limit and the location of the metal single atom are discussed, combining experiments with simulations. In addition, we demonstrate that the coordination structure of the metal single atom can be tailored to address the relationship of structure and performances of the metal SAC in reactions. We expect that this perspective can provide some insights to guide the study for the rational design of thermally-stable and active single atom catalysts, which are especially suitable for high-temperature reactions.

## Introduction

Catalysis has been in the era of the precise design and manipulation of catalyst structure in the atomic scale for developing highly efficient catalysts (Guan et al., 2021). Single-atom catalysis has attracted extensive attention since it was proposed by Zhang et al., in 2011 (Qiao et al., 2011) in that it can bridge the gap between homogeneous catalysis and heterogeneous catalysis. Because of the high atom efficiency, single-atom catalysts (SACs) have therefore attracted ever-increasing attention from numerous fields including material science, catalysis and electrochemistry. To date, much progress has been achieved on the studies of metal SACs in catalysis, especially on the synthesis and characterization of metal SACs (Li et al., 2018; Ji et al., 2020). Furthermore, metal SACs have been found to present superior reactivity (selectivity or activity) than nanoparticles in several catalytic reactions, such as hydrogenation (Yan et al., 2015) and oxidation (Zhang et al., 2022a). However, most of these reactions were carried out at relatively low reaction temperatures (<100°C) and catalytic reactions performed at temperatures of >200°C, such as dehydrogenation and reforming, are rarely reported since metal SACs are thermodynamically unstable and are prone to agglomerate at elevated temperatures due to Ostwald ripening (OR).

Metal SACs must keep stable during chemical reactions under industrial conditions, including at elevated temperatures (Xiong et al., 2021a). Especially, in the transition from the academic curiosity to an industrially relevant technology, the thermal stability of metal SAC became much more important (Datye and Guo, 2021). Previous work has indicated that metal SACs prepared by atom trapping (AT) can withstand the temperature up to 800°C in oxidizing conditions (Jones et al., 2016; Lang et al., 2019). However, many metal SACs are not stable under reaction atmospheres or at elevated temperatures. These SACs have been demonstrated to agglomerate to form nanoclusters due to the high free energy of SACs under reaction conditions (Yang et al., 2013). For example, atomically dispersed metal atoms can rapidly agglomerate to metal clusters or nanoparticles under catalytic reactions (CO oxidation, hydrogenation and dehydrogenation) (Liu et al., 2019). Moreover, the size of Pt particles formed from single atoms on a Pt/Al_2_O_3_ increases with the reaction temperature from 150 to 325°C, indicating that Pt species undergo dynamic structural transformation during reaction (Liu et al., 2019). Therefore, the development of metal SACs that are stable under reaction conditions is pivotal, which is prerequisite for future commercialization of these catalysts (Datye and Guo, 2021).

In this perspective, we discuss the progress on the preparation and activation of thermally-stable single-atom catalysts (TSSAC) in catalysis. We firstly introduce atom trapping (AT) and vapor-phase self-assembly (VPSA) to prepare thermally stable single atom catalysts, including on the supports of ceria (CeO_2_) and MgAl_2_O_4_. The ceria represents the supports with strong metal-support interaction, while the MgAl_2_O_4_ represents the supports with weak metal-support interaction. We also describe two approaches to tailor the coordination structure of the Pt single atoms on the thermally-stable Pt_1_/CeO_2_ catalyst. Finally, the atom-trapped Pt_1_/CeO_2_ SAC can be used to load a second metal atoms to generate two-dimensional metal oxides which shows superior catalytic reactivity than three-dimensional metal oxides. For the general and comprehensive understanding of SAC or TSSAC, such as support choices or carbon-supported SAC, the readers are referred to other important review articles (Liu et al., 2019; Xiong et al., 2021a; Singh et al., 2021).

## Atom trapping for the preparation of TSSAC

Metal atoms in nanoparticles are mobile at high temperatures, leading to the sintering of the nanoparticles *via* the Ostwald Ripening mechanism. The mobile atom can be trapped by oxide supports such as PdO (Xiong et al., 2016), CeO_2_ (Jones et al., 2016; Wan et al., 2018) and Fe_2_O_3_ (Lang et al., 2019) or carbon materials (Wei et al., 2018) to form single-atom catalysts (Figures 1A,B). The trapping of the mobile metal atom by CeO_2_ and Fe_2_O_3_ is due to the strong metal atom-support interaction. In 2016, we first reported the evaporated migration of Pt species from Pt nanoparticles on alumina to ceria surface *via* a reverse Ostwald ripening mechanism (Jones et al., 2016). The Pt species was then trapped by the ceria and located on the ceria surface to form Pt_1_/CeO_2_ SAC. Further study found that the Pt1/CeO_2_ SAC can be formed by directly dispersing Pt salt precursors onto the ceria, followed by annealing the material at elevated temperatures in air. The locations and the maximum loading of the Pt single atom on the polyhedral ceria was further investigated (Kunwar et al., 2019). It is demonstrated that cerium oxide supported Pt single atoms at high metal loading up to 3 wt.% Pt. This Pt loading corresponds to the maximum density of Pt single atom on the ceria surface is ca. 1 Pt atom/nm^2^.

**FIGURE 1:** Atom trapping for the preparation of thermally-stable Pt single atom catalysts. **(A)** Illustration of Pt nanoparticle sintering and redispersion. Reproduced with permission (Jones et al., 2016). Copyright 2016, American Association for the Advancement of Science. **(B)** Illustration of the redispersion of Pt nanoparticle to Pt single atoms on Fe_2_O_3_. Reproduced with permission (Lang et al., 2019). Copyright 2019, Springer Nature. **(C)** Schematic illustration of the vapor-phase self-assembly processes. **(D)** AC-STEM image of Pt/K/MgAl_2_O_4_ SAC. **(E)** Catalytic reactivity and stability of Pt catalysts. **(F)** Reactivity and stability of Pt/K/MgAl_2_O_4_ SAC and Pt/MgAl_2_O_4_ nanocatalyst in methane oxidation. Reproduced with permission (Li et al., 2022). Elsevier.

The catalytic reactivity of the Pt_1_/CeO_2_ SAC prepared by the high temperature vapor phase synthesis (atom trapping, AT) was compared with Pt_1_/CeO_2_ SAC prepared by conventional wetness synthesis (strong electrostatic adsorption-SEA) with calcination at 350°C in air in CO oxidation (Pereira-Hernández et al., 2019). The AT sample led to ionic Pt being trapped on the CeO_2_ in a thermally stable form. The as-synthesized, both SACs are inactive for low- temperature (<150°C) CO oxidation. After treatment in CO at 275°C, both catalysts show enhanced reactivity. Despite similar Pt metal particle size, the AT catalyst is significantly more active, with onset of CO oxidation near room temperature. A combination of near-ambient pressure X-ray photoelectron spectroscopy (NAP-XPS) and CO temperature-programmed reduction (CO-TPR) showed that the high reactivity at low temperatures was related to the improved reducibility of lattice oxygen on the CeO_2_ support.

## Vapor-phase self-assembly for the preparation of TSSAC

For the oxide supports with a weak metal-support interaction such as Al_2_O_3_ and MgAl_2_O_4_, experiment results showed that these oxide supports could not directly trap the mobile metal atom to form single-atom catalyst at high temperatures. Instead, the mobile metal atoms agglomerated to form large particles due to sintering at elevated temperatures (Xiong et al., 2016). Recently, an approach termed as “vapor-phase self-assembly” was reported to trap the mobile metal single atoms on the support having a weak metal-support interaction (Li et al., 2022). The new design principle, efficiently anchored Pt single atoms on a conventional support MgAl_2_O_4_ with the assistant of K ions at elevated temperature in air. A stable triangular K_3_O_3_ structure serves as sites for trapping isolated Pt species over MgAl_2_O_4_ (111), leading to a superior stability in methane oxidation. Such Pt single atoms trapped by the triangle motif are capable of withstanding exposure to high temperatures in oxidizing conditions. The Pt/K/MgAl_2_O_4_ SAC presented excellent thermal/hydrothermal stability and reactivity in methane oxidation in the presence of steam at elevated temperatures (Figures 1C–F), as compared to the Pt/MgAl_2_O_4_ nanocatalyst without K and the Pt_1_/CeO_2_ SAC.

The generalizability of the vapor-phase self-assembly mechanism on stabilizing metal single atoms was investigated on other alkali metal cations, metal centers and oxide supports. Alkali metal cations of Li^+^, Na^+^ and Cs^+^, metal centers (Ru, Ir and Au) and oxide supports (SiO_2_, NiAl_2_O_4_, CoAl_2_O_4_ and MgCr_2_O_4_) as well as density functional theory (DFT) simulations were used to explain the different effects of these structural parameters on stabilizing the metal single atoms during the VPSA process. Results show that alkali Na^+^ and Cs^+^ can stabilize the Pt single atoms on MgAl_2_O_4_ after the VPSA, whereas Li^+^ cannot trap Pt single atoms. DFT simulations revealed that for the Na^+^, K^+^ and Cs^+^, the atoms in the M-O motifs (M = Na, K and Cs) are in the same plane, while the atoms of Li-O motif in the *Z* direction are not in the same plane, leading to a weak interaction between Li and O on MgAl_2_O_4_ (111). As for other metal single atoms (Ru, Ir and Au), the K-modified MgAl_2_O_4_ can stabilize Ru and Ir atoms with VPSA, while it cannot stabilize Au atom. DFT calculations showed that after depositing M_1_, a stable triangle M_1_O_3_ structure is formed for Ru and Ir, similar to the case of Pt_1_ single atom. For oxide supports, *γ*-Al_2_O_3_ cannot trap Pt single atoms *via* VPSA because of the irregular surface revealed by DFT simulation, which cannot stabilize KO motif. The K/NiAl_2_O_4_ and K/CoAl_2_O_4_ cannot trap the Pt single atoms, whereas K/MgCr_2_O_4_ can partially trap the mobile Pt atoms at elevated temperatures. DFT simulations confirm the above observations.

## Modulation of the coordination structure of TSSAC

Pt_1_/CeO_2_ SAC prepared by AT is thermally stable, while it is not as active as Pt/CeO_2_ nanocatalyst in CO oxidation (Gänzler et al., 2017; Pereira-Hernández et al., 2019). This is because the Pt single atom on the AT sample was strongly bound on the ceria. To improve the reactivity of the Pt_1_/CeO_2_ SAC, the coordination environment of the Pt single atom must be tailored. Two strategies were reported to modulate the coordination structure of the Pt single atom in the Pt_1_/CeO_2_ SAC. One is the addition of a second metal atom into the Pt_1_/CeO_2_ SAC (Xiong et al., 2017), such as Sn or Ga. The reactivity and stability of Pt single-atom species was investigated in the industrially important light alkane dehydrogenation reaction. The Pt_1_/CeO_2_ single-atom catalyst is active during propane dehydrogenation, but not selective for yielding propylene. DFT calculations show strong adsorption of the olefin produced, leading to C-C cleavage to produce CH_4_. In contrast, the addition of tin (Sn) into Pt_1_/CeO_2_ SAC allows the modified SAC to achieve high selectivity towards propylene because of facile desorption of the product. Furthermore, upon oxidation the Pt-Sn species readily revert to the atomically dispersed species on CeO_2_, making Pt-Sn/CeO_2_ a fully regenerable catalyst. Ga was also used to modify the coordination structure of the Pt_1_/CeO_2_ SAC in CO oxidation (Feng et al., 2018). Significantly, the stability of Pt single atoms anchored on the Ga site was enhanced compared with those on the bare ceria surface.

The other approach used to modify the coordination structure of Pt_1_/CeO_2_ SAC is to treat the Pt_1_/CeO_2_ SAC in a high-temperature steam (750°C) (Nie et al., 2017). The results demonstrated that the Pt_1_/CeO_2_ was activated *via* steam treatment (at 750°C) to simultaneously achieve the low-temperature CO oxidation activity while keeping Pt atomically dispersed after the high-temperature steam treatment. The treated Pt_1_/CeO_2_ SAC reached 100% CO conversion at 150°C, as compared to the inactive Pt_1_/CeO_2_ SAC at the same temperature in CO oxidation. A new type of active site is created on CeO_2_ in the vicinity of Pt^2+^, where Pt cation is coordinated with O_lattic_H to provide the improved reactivity in the oxidations of CO, NO and propane. These active sites are stable up to 800°C in oxidizing environments.

## Engineering catalyst support *via* TSSAC

Metal single atoms in SAC can be used to engineer the properties of the support surface. Relying on the trapping of Pt single atoms on the CeO_2_ surface in thermally stable form, the nature of the deposited metal/metal oxide clusters can be modified (Xiong et al., 2021b). In particular, two-dimensional (2D) rafts of PtO_x_ on the engineered catalyst support are formed by this approach (Figures 2A–C), as opposed to three-dimensional (3D) metal oxide nanoparticles on conventional supports. This 2D rafts of PtO_x_ showed much higher reactivity than a Pt_1_/CeO_2_ SAC and the 3D Pt/CeO_2_ catalyst in CO oxidation (Xiong et al., 2021b). Adopting this approach for the synthesis of bimetallic catalysts *via* addition of Pd to the atom-trapped catalyst support (Pt@CeO_2_), the resulting Pd/Pt@CeO_2_ catalyst (Figures 2D–F) provides three times higher reaction rate and improved water tolerance than an impregnated PtPd/CeO_2_ catalyst during methane oxidation. The improved performance is attributed to the 2D morphology of the PdO_x_ phase presented on the atom-trapped Pt@CeO_2_ support. The results showed that modifying the support by trapping single atoms provided an important addition to the toolkit of catalyst designers to engineer catalyst supports for controlling the nucleation and growth of metal and metal oxide clusters in heterogeneous catalysts.

**FIGURE 2:** Engineering catalyst support *via* thermally-stable single-atom catalyst. **(A)** Schematic illustration showing the morphologies of Pt catalysts supported on ceria prepared by depositing Pt on a Pt-trapped ceria (Pt@CeO_2_) **(B,C)** AC-STEM images of the catalyst prepared by depositing 2 wt.% Pt on atom-trapped 1 wt.% Pt@CeO_2_. **(D,E)** AC-STEM image of Pd deposited on the catalyst shown in **(E)**. **(F)** Comparison of catalyst stability for the as-synthesized 1Pd/2Pt@CeO_2_ and (1Pd + 2Pt)/CeO_2_ catalysts, reduced 2Pt@CeO_2_ and reduced 1Pd/CeO_2_ catalysts in CH_4_ oxidation at 500°C in 4% H_2_O. Reproduced with permission (Xiong et al., 2021b). Copyright 2021, Springer Nature.

## Summary and perspective

To summarize, single-atom catalysts (SACs) are promising because of their maximum atom efficiency and unique property in catalysis. However, recent studies demonstrate that metal SACs tend to sinter to form clusters under reaction conditions, especially at elevated temperatures. Considering many catalytic reactions such as dehydrogenation, syngas chemistry and reforming, are carried out at temperatures of >200°C, it is therefore important to develop approaches to prepare thermally stable and active SACs for their future commercialization. In this perspective, the preparation and catalytic application of thermally-stable metal SACs are summarized, mainly on Pt-based SACs. *Via* the reverse-Ostwald ripening mechanism, approaches including atom trapping and vapor-phase self-assembly were applied to prepare stable and active Pt SACs. The locations of the Pt single atoms on the supports (CeO_2_ and MgAl_2_O_4_) were also corroborated using both experiments and simulations, and the properties of the Pt SACs were well demonstrated by advanced techniques such as XAS, LEIS, AC-STEM and CO-DRIFTS. In addition, the coordination environment of the metal SACs was tailored by different approaches such as adding the second metal or treating SAC in high-temperature steam. We also discuss the engineering of the catalyst support by atom-trapped single atoms, which modified the morphology of the deposited metal/metal oxide to achieve unique catalytic performances in catalysis.

Metal SAC used in practical catalytic reactions must be thermally stable under realistic conditions and therefore this area will unambiguously attract continuing attention in future. Focusing on thermally stable and active metal SACs, we would like to provide our insights on the future studies in this field. Firstly, metal SAC that is stable under oxidizing conditions may be not stable under reducing conditions, especially at elevated temperatures. Future work needs to perform to improve the catalyst stability under reducing conditions at elevated temperatures. Secondly, not all stable metal SACs are active or selective in catalysis. Therefore, the coordination structure of the metal single atom needs to be tailored to improve the activity/selectivity. Although there are a couple of strategies reported to adjust the coordination structure of metal center, a general approach applicable to other metal SACs is lacking. Thirdly, photocatalysis and electrocatalysis have attracted the ever-increasing interests in catalysis because these energies are renewable, and the use of these energies have the potent to go net zero. Since noble metal catalysts are widely used in these processes (Zhang et al., 2022b), photo-/electro- stability of metal single-atom catalysts suitable for both photocatalysis and electrocatalysis is therefore worthy investigating. Finally, current studies on metal SACs are mostly tested in several model reactions, including CO oxidation, semi-alkyne hydrogenation and the preferential oxidation of CO (PROX). The temperatures in these reactions are relatively low. Therefore, the stability of metal SACs must be examined in other conventional reactions such as syngas conversion and reforming, where a couple of recent studies have pioneered in this field recently (Akri et al., 2019; Tang et al., 2019).

## Data Availability

The original contributions presented in the study are included in the article/Supplementary material, further inquiries can be directed to the corresponding author.
